The article "Detecting Cognitive Impairment Status Using Keystroke Patterns and Physical Activity Data among the Older Adults: A Machine Learning Approach" was published in 2021. Journal: J Healthc Eng.

# Detecting Cognitive Impairment Status Using Keystroke Patterns and Physical Activity Data among the Older Adults: A Machine Learning Approach

**DOI:** 10.1155/2021/1302989

**Published:** 2021-12-20

**Authors:** Mohammad Nahid Hossain, Mohammad Helal Uddin, K. Thapa, Md Abdullah Al Zubaer, Md Shafiqul Islam, Jiyun Lee, JongSu Park, S.-H. Yang

**Affiliations:** ^1^Department of Electronic Engineering, Kwangwoon University, Seoul 139-701, Republic of Korea; ^2^Smart H&B Technology Laboratory, Department of Electronic Engineering, Kwangwoon University, Seoul 139-701, Republic of Korea

## Abstract

Cognitive impairment has a significantly negative impact on global healthcare and the community. Holding a person's cognition and mental retention among older adults is improbable with aging. Early detection of cognitive impairment will decline the most significant impact of extended disease to permanent mental damage. This paper aims to develop a machine learning model to detect and differentiate cognitive impairment categories like severe, moderate, mild, and normal by analyzing neurophysical and physical data. Keystroke and smartwatch have been used to extract individuals' neurophysical and physical data, respectively. An advanced ensemble learning algorithm named Gradient Boosting Machine (GBM) is proposed to classify the cognitive severity level (absence, mild, moderate, and severe) based on the Standardised Mini-Mental State Examination (SMMSE) questionnaire scores. The statistical method “Pearson's correlation” and the wrapper feature selection technique have been used to analyze and select the best features. Then, we have conducted our proposed algorithm GBM on those features. And the result has shown an accuracy of more than 94%. This paper has added a new dimension to the state-of-the-art to predict cognitive impairment by implementing neurophysical data and physical data together.

## 1. Introduction

Cognitive impairment, also known as neurocognitive disorders, is a loss of cognitive function. It has destructive effects on people and the community as well. People with this condition have problems with perception, attention, and memory; meanwhile, these are essential things to build human cognition and psychiatric disorders (e.g., depression, insomnia, psychotic symptoms, etc.) [1–3] and even physical diseases, such as diabetes mellitus (DM) and cardiovascular diseases [4]. People with cognitive impairment also experience a diminished quality of life [5].

Cognitive impairment can cause many psychological symptoms in patients [6]. Its devastating consequences may increase the risk of dementia [7]. A study has shown that about 30–40% of cases with cognitive impairment subsequently progress to dementia [8]. The total assessed expense of dementia was US$818 billion in 2015, implying 1.09% of worldwide total domestic product [9]. The economic difficulty and pathological complexities among victims with cognitive impairment are undoubtedly more crucial [10]. Researchers have figured out that by 2030, people with dementia will be about 75 million, and this contingency will cost the community US$ 2 trillion [11]. Early detection of cognitive impairment status supports a sufferer by allowing them to plan for the future and early treatment [12–14].

The article "Detecting Cognitive Impairment Status Using Keystroke Patterns and Physical Activity Data among the Older Adults: A Machine Learning Approach" was published in 2021. Journal: J Healthc Eng.

At present, an ideal approach to confine or limit this overwhelming course is identifying danger in individuals and starting intervention early [15]. Many researchers have explored neurobiological, hereditary, EEG signal, and neuroimaging biomarkers for cognitive impairment diagnosis, especially in Alzheimer's disease [15, 16] and also dementia [17]. Magnetic resonance imaging (MRI) [18] and neuroimaging techniques were broadly used to detect cognitive impairment [19–21]. Many AI-inspired approaches have been discovered, yet no quantitative analysis of accomplishment is proposed. AI approaches using machine learning, artificial neural network, and deep learning show some significant improvement in impairment detection but still have challenging issues.

We have proposed an advanced ensemble learning algorithm named Gradient Boosting Machine (GBM) to detect cognitive impairment among older adults. Data obtained from the smartwatch and keystroke were preprocessed and analyzed through Pearson's correlations. Then, the wrapper feature selection technique was used to select the best features. Experimented algorithms were chosen by observing the distribution (standard deviation, outliers, etc.) of our dataset. The selective features have been trained and tested with proposed algorithms to determine the best prediction results. Our proposed method highlights the following:

1. We have proposed a combination of physical and neurophysical data to detect cognitive impairment levels.
2. A conventional customized machine learning technique is performed to detect cognitive impairment, and classification performances are compared with other models.
3. The accuracy is higher for this quantitative analysis of detecting cognitive impairment.
4. In particular, our proposed method has the best accuracy of predicting mild cognitive impairment (MCI) than previous work.

The health care services area is perhaps the leading region for AI applications. It is quite possibly the most complex field [22] and may be the most testing, particularly in the areas of conclusion and expectation [23]. Given that early mediation can decrease cognitive deterioration, current cognitive appraisals can be ineffective and develop older adults' technology use. So, our proposed methodology can make a turnover to lead a happy life for older adults.

The article "Detecting Cognitive Impairment Status Using Keystroke Patterns and Physical Activity Data among the Older Adults: A Machine Learning Approach" was published in 2021. Journal: J Healthc Eng.

## 2. Related Works

There are many kinds of research ongoing on the prediction of cognitive impairment using simple-to-deep learning algorithms. Artificial neural network (ANN) algorithm has been used to distinguish the cognitive state using multicenter neuropsychological test data with magnificent accuracy [24]. Reference [24] was confined to neuropsychological tools for diagnosing cognitive impairment. Random forest survival analysis and semiparametric survival analysis (Cox proportional hazards) were combinedly used to evaluate the relative significance of 52 predictors in predicting cognitive impairment and dementia immensely [25]. Reference [25] was time-consuming research, having some limitations. One is that predictive correlations were focused on correlational analysis, which is implicitly bidirectional. The other is that cognitive outcome calculations were based on a success index for self-respondents and a ranking measure for proxy respondents rather than on clinical diagnosis. Artificial Intelligence (AI) approaches, including supervised and unsupervised machine learning (ML), deep learning, and natural language processing, have been applied for cognitive impairment by providing a conceptual overview of this topic, emphasizing the features explored [26]. A more effective method has been experimented for monitoring cognitive function using keystrokes [27] and linguistic characteristics with IT [28]. There are some limitations mentioned that should be solved, like security concerns about providing personal data. The “Panoramix suite-6” serious digital games (“Episodix,” “Attentix,” “Semantix,” “Workix,” “Procedurix,” and “Gnosix”) scores datasets have been experimented through some renowned ML (SVM, CART, and LR) algorithms to detect cognitive impairment [29]. But it may discriminate in result when targeting older adults. Based on the b test's accuracy, a model has been developed to detect cognitive symptoms malingering in predicting malingerers of mild cognitive impairment [30]. This research was based on the medical symptoms of patient datasets. These models' applicability has spread in different directions [31, 32]. Magnetic resonance imaging (MRI) [33], in combination with multiplex neural networks [34], and resting-state functional magnetic resonance imaging (rs-fMRI), in combination with graph theory [35], have been used to isolate healthy brains from progressive mild cognitive impairment (pMCI), in the diagnosis of AD and MCI. These researches were based on functional data. When applied to functional data from groups of healthy control subjects and MCI and AD patients, AD and MCI could be identified as induced causes to the brain network. Based on the cognitive neuroscience researchers' abnormal activity routines datasets, a novel hybrid statistical-symbolical technique can detect cognitive impairment [36]. This study achieved promising results. But the recognition method was based on only nonprobabilistic rules that strictly determine the detection of an abnormal behavior based on a user-defined set of observations. Besides, based on routine primary care patient datasets, conventional statistical methods and modern machine learning algorithms have been used to develop a risk score [37] to determine how people may build dementia [38]. Few research studies have been published where a systematic [39], quantitative, and critical review [40] has been analyzed to predict cognitive impairment and dementia using different machine learning techniques. Few research studies have also developed machine learning algorithms to detect cognitive impairment based on authorized clinical questionnaires' datasets only [41, 42].

The article "Detecting Cognitive Impairment Status Using Keystroke Patterns and Physical Activity Data among the Older Adults: A Machine Learning Approach" was published in 2021. Journal: J Healthc Eng.

## 3. Materials and Method

This study aims to develop a model for classifying cognitive impairment levels using keystroke patterns and physical activity information.  Figure 1 represents a flowchart describing the whole development of the system, which consists of four phases. In the data collection phase (Figure 1(a)), three types (keystroke patterns, physical, and SMMSE score) of data have been collected. In the data collection phase, keystroke patterns data as neurophysical data are collected from a developed android application. Regular physical activity data is collected from smartwatches, and SMMSE data is collected from the questionnaire session, as shown in Figure 1(a). After extracting features, feature analysis has been performed to determine the correlations in features and then select the highly correlated features, as shown in Figure 1(b). After Analyzing the dataset feature, a machine learning algorithm has been chosen, as shown in the machine learning approach phase (Figure 1(c)). The result analysis phase has demonstrated the relation between features output and SMMSE score output using the regression model and showing the validation using “10-fold cross-validation” (Figure 1(d)).

Participants' mental health status in terms of cognitive impairment has been assessed using the twelve-item Standardised Mini-Mental State Examination (SMMSE). The British Columbia Ministry of Health validates this SMMSE approach, and the questionnaire can also be found on their website [43]. Several research types [44–47] used these questions for related cognitive issues. For this study, we also selected these questions, and 33 participants were asked SMMSE questions to generate the SMMSE score. This score represents the cognitive impairment's actual value to label the participant for group selection. There are 26 males and seven females whose age range is between 50 and 65. They were followed up for up to 6 months. In this study, the participant's cognitive impairment levels have been categorized into four types based on SMMSE score: normal (SMMSE score ≥  25), mild (21 ≤ SMMSE score ≥ 24), moderate (10 ≤ SMMSE score ≥ 21), and severe (SMMSE score ≤ 9).  Table 1 represents the distribution of the cognitive impairment scores based on the SMMSE. Every day, SMMSE scores were collected from participants. Some data were excluded because of insufficient information.  Table 2 represents a sample of our datasets.

The article "Detecting Cognitive Impairment Status Using Keystroke Patterns and Physical Activity Data among the Older Adults: A Machine Learning Approach" was published in 2021. Journal: J Healthc Eng.

### 3.1. Data Collection

We have collected the datasets from the Bangladesh research organization. The study's motive was to detect cognitive impairment via keyboard stroke patterns and activities they performed every day, such as sleeping, walking, etc. This study's data is collected using smart environment technologies, including android applications and wearable smartwatches.

On a particular day, the participant came to the research center smart apartment and performed keyboard stroke patterns activity, and this neurophysical data was recorded. Physical data were collected from the smartwatch they wore all day long. Also, the SMMSE score was generated through a questionnaire session.

Participants were assigned identifiers during the study. The identifiers have been randomized before this data was made available to the research.

### 3.2. Data Preprocessing

#### 3.2.1. SMMSE Score Estimation

The SMMSE score has been taken at the beginning of the study and represents the participant's cognitive impairment severity. The presented study explores each extracted feature correlated with cognitive impairment symptoms that can differentiate participants from cognitive impairment. This questionnaire score was estimated by using a linear regression model [48] on extracted features. The standard linear regression model can be represented as follows:

(1) $$\begin{array}{c} {\bar{E}}_{\text{iesmmse}}=\alpha_{0}+\alpha_{1}f_{1}+\alpha_{2}f_{2}+\cdots +\alpha_{n}f_{n}, \end{array}$$

where *Ē*_iesmmse_ is the estimated score of SMMSE for *i*th participants, *f*_*n*_ is the *n* number of features, and *α*_0_, *α*_1_, *α*_2_, ...,  *α*_*n*_ are the coefficients of the linear regression model.

The article "Detecting Cognitive Impairment Status Using Keystroke Patterns and Physical Activity Data among the Older Adults: A Machine Learning Approach" was published in 2021. Journal: J Healthc Eng.

The lasso regularization [49] was used to minimize the error between the estimated score and the actual SMMSE score. The lasso regularization restricted the regression model coefficient to become too high. It performed well in the model as all the features were highly correlated.

(2) $$\begin{array}{c} {\bar{E}}_{lr}=\sum_{i=1}^{n}{\left(y_{i\;}-\sum_{j}x_{ij}\beta_{j}\;\right)}^{2}+\lambda \sum_{j=1}^{p}\left|\beta_{j}\right|, \end{array}$$

where *Ē*_lr_ is the lasso regularization. The first part of equation (2) represents the “residual sum of squares,” and the other part represents as the “sum of the absolute value of the magnitude of coefficients,” and *λ* denotes the amount of shrinkage.

#### 3.2.2. Data Augmentation

The class imbalance may damage the predictive model's performance, most of the time, in machine learning algorithms because machine learning algorithms focus more on detecting the larger classes. Our dataset has class imbalance problems, which suggest that the predictive models could poorly detect the minority class. We have tried to mitigate the class imbalance problem by augmenting 10% of our datasets' data using the Conditional Tabular GAN (CTGAN) [50] algorithm with high fidelity. CTGAN is another GAN designed to synthesize tabular data proposed in 2019 by the same authors as TGAN [51]. As shown in Figure 2, the statistical descriptions between original data and augmented data have been given. Every value like mean, standard deviation, minimum, and maximum into original and augmented data is almost the same. It indicates that, after augmentation, the distributions of datasets remain the same.

### 3.3. Feature Extraction

A total of 11 features have been extracted from participants' classified neurophysical behavior and physical activity patterns information. Four features for neurophysical behavior from our developed application and another seven physical activity features from wearable devices are shown in Table 3.

### 3.4. Feature Subgroup

Our analysis has explored that working and nonworking day's features have some relationship based on the extracted features of days. So, we have divided our extracted features into three subgroups: (i) baseline, (ii) weekdays, and (iii) weekend days.

(3) $$\begin{array}{c} {\bar{E}}_{n}=\sum_{i=1}^{n}D_{i}. \end{array}$$

In the equation, *Ē*_*n*_ represents the feature subgroup, *n* is the total number of days based on feature subgroups: baseline, *n* = 7; weekdays (Sunday to Thursday), *n* = 5; and weekend days (Friday and Saturday), *n* = 2. *D*_*i*_ represents the *i*th day features.

### 3.5. Feature Selection

Feature selection is a strategy to choose optimal features from datasets. This technique improves model performance and reduces complexity and computational costs. Also, it can improve the accuracy, reduce the overfitting, speed up training, improve data visualization, and increase the explainability of the model. In this study, we have used the Pearson correlation coefficient [53] to analyze the feature. Pearson's correlation coefficient formula is

(4) $$\begin{array}{c} r=\frac{\sum \left(x_{i}-\underline{x}\right)\left(y_{i}-\underline{y}\right)}{\sqrt{\sum {\left(x_{i}-\underline{x}\right)}^{2}-\sum {\left(y_{i}-\underline{y}\right)}^{2}}}, \end{array}$$

where *r* is the correlation coefficient, *x*_*i*_ is the *x*-variable in a sample, $\underline{x}$ is the mean of the values of the *x*-variable, *y*_*i*_ is the values of the *y*-variable in a sample, and $\underline{y}$ is the mean of the values of the *y*-variable.

The article "Detecting Cognitive Impairment Status Using Keystroke Patterns and Physical Activity Data among the Older Adults: A Machine Learning Approach" was published in 2021. Journal: J Healthc Eng.

Using Pearson's correlation, we can generate an “*r*” value of individual features to rank the datasets' significant features. This “*r*” value can vary between −1 and 1.  Figure 3 shows the total scenario of every feature's correlation with each other. The “*p*” value also plays a significant role in choosing the features.  Figure 4 shows the correlation with each other based on “*p*” values. If this “*p*” value of any feature is less than 0.05 and near to 0, that feature would be a significant feature. Our analysis has been shown from the “*r*” values heatmap and the “*p*” values heatmap. As shown in Figures 3 and 4, we can observe that some features are highly correlated, while some features are less correlated. It indicates that some features would be significant, and some would not be so for our model.

Then, the wrapper feature selection method [54] has been used to select the model's best features. Regression and a classification algorithm have been used to evaluate the selected feature's performance after “10-fold cross-validation” of the data. Regression model features have been selected using the root mean square deviation (RMSD) of the SMMSE score estimation.

### 3.6. Methods

Cognitive impairment was classified into four categories (Table 3), and for evaluating the classification performance, we mainly focus on supervised learning. Two famous classification algorithms, Ensemble Learning (EL) and Support Vector Machine (SVM), were considered to detect the users' cognitive impairment.

#### 3.6.1. Gradient Boosting Machine (GBM)

The Gradient Boosting Machine (GBM) [55] algorithm is an advanced algorithm of Ensemble Learning (EL) algorithm. It is a supervised machine learning algorithm for regression and classification problems. It generates a prediction model, commonly decision trees. Meanwhile, a decision tree is a weak learner, and the resulting algorithm is called gradient boosted trees, which usually outperforms random forest. It creates the model sequentially as other boosting techniques do. Then, subsequence models are trying to reduce the error of the previous model. Each model reduces the error of the previous model by building the model on the error of residuals of the previous prediction. This is done to determine if there are any patterns in the errors that the previous model missed. And we repeat the same process: either the error becomes zero or we have reached the stopping criteria, which is the limit to the number of models we have built. Then, it concludes them by allowing optimization of an absolute differentiable loss function. We have given GBM working procedures step by step in a block diagram as shown in Figure 5. In a nutshell, we built our first model, which has features *x* and target *y*. And the first model was named *H*_0_, which is a function of *x* and *y*. Then, we built the next model on the error of the previous model repeatedly till the *n*th model, as shown in Figure 6.

The article "Detecting Cognitive Impairment Status Using Keystroke Patterns and Physical Activity Data among the Older Adults: A Machine Learning Approach" was published in 2021. Journal: J Healthc Eng.

*H*_0_ gives some predictions and generates error *e*_0_ by the function “*F*_0_ (*X*)” as shown in equation (4). Then, the next model added the new predicted errors *e*_1_ with “*F*_0_ (*X*)” creating a new function “*F*_1_ (*X*)” as shown in equation (5). Similarly, we built the next model as shown in equation (6) till the *n*th model.

(5) $$\begin{array}{c} F_{0}\left(X\right)=\gamma_{0}H\left(x,y\right)+e_{0}. \end{array}$$

(6) $$\begin{array}{c} F_{1}\left(X\right)=F_{0}\left(X\right)+\gamma_{1}H_{1}\left(X,e_{0}\right)+e_{1}. \end{array}$$

(7) $$\begin{array}{c} F_{2}\left(X\right)=F_{1}\left(X\right)+\gamma_{2}H_{2}\left(X,e_{1}\right)+e_{2}, \end{array}$$

and the final equation is something like that shown in equation (7). In equation (7), “*F*_*n*-1_ (*X*)” is the prediction by the previous model. Some new predicted errors were added to this model. Finally, we are left with some errors named *e*_*n*_. So, at every step, we are trying to model the errors that help us reduce the overall error, and our focus is that the error tends to be zero (i.e., *e*_*n*_ = 0). Each model here is trying to boost the performance of the model. We add a coefficient “*γ*” and the proper value of this coefficient will be decided using the gradient descent technique.

(8) $$\begin{array}{c} F_{n}\left(X\right)=F_{n-1}\left(X\right)+\gamma_{n}H_{n}\left(X,e_{n-1}\right)+e_{n}. \end{array}$$

The generalized equation will be like that shown in equation (8). It represents “*F*_*n*_ (*X*)” as all the previous models, *γ*_*n*_ represents the coefficient, and “*H*(*X*, *e*_*n*_)” the current working model function, where *X* represents the features and *e*_*n*_ means the model's error.

(9) $$\begin{array}{c} F_{n+1}\left(X\right)=F_{n}\left(X\right)+\gamma_{n}H\left(X,e_{n}\right). \end{array}$$

If we dive deeper into equation (9), to understand about loss function and calculate *γ*_*n*_. We consider a loss function as shown in equation (10) where *y* is the actual value and *y*′ is the predicted value for the last model. So, the square difference of this would be the loss.

(10) $$\begin{array}{c} L={\left(y-y^{\prime }\right)}^{2}. \end{array}$$

In our case, the target here is *y*, where *y*′ can be considered the updated prediction of the last model. So, we can replace *y*′ with *F*_*n*_ (*X*), and the new equation will be as follows:

(11) $$\begin{array}{c} L={\left(y-F_{n}\left(X\right)\right)}^{2}. \end{array}$$

Here, we will use gradient descent techniques and differentiate this equation (10) with respect to *F*_*n*_(*X*). We will get something like that shown in the following equation:

(12) $$\begin{array}{c} \frac{\text{d}L}{\text{d}F_{n}\left(X\right)}=-2\left(y-F_{n}\left(X\right)\right). \end{array}$$

To simplify this equation (12), we will multiply both sides with “−1”. And we will get something like that shown in the following equation:

(13) $$\begin{array}{c} -\;\frac{dL}{dF_{n}\left(X\right)}=2\left(y-F_{n}\left(X\right)\right). \end{array}$$

Now the right-hand side of the equation is similar to the error we are discussing. Here, we consider the error *e*_*n,*_ which is actually (*y* − *F*_*n*_(*X*)). So, it can be said that *e*_*n*_ is also equal to the left-hand side of the equation. So, it can be replaced, that is, *H*(*X*, −*dL*/*dF*_*n*_(*X*)), and our final equation will be as follows:

(14) $$\begin{array}{c} F_{n+1}\left(X\right)=F_{n}\left(X\right)+\gamma_{n}H\left(X,-\frac{dL}{dF_{n}\left(X\right)}\right). \end{array}$$

Now the aim is to minimize the overall loss function. So, the overall loss would be the loss we get from all the models we have built so far, as shown in the following equation:

(15) $$\begin{array}{c} \text{LOSS}=L\left(y,F\left(X\right)\right)+\gamma_{n}L\left(H\left(X,-\frac{dL}{dF_{n}\left(X\right)}\right)\right). \end{array}$$

The first part of the overall loss is fixed as these are the predictions we have generated from the previous models we built. So, this cannot be changed. The second part of this equation has another loss of the current model, and this loss cannot be changed. But we can still change the gamma value. Now it needs to select a value of gamma such that the overall loss is minimized. And this value would be selected using a gradient descent process. The idea is to minimize the overall loss by deciding the right value of gamma for each model. So, the next model, when we built that model, will again have the coefficient of *γ*_*n*_, and we try to select the right value such that the overall loss is minimum. For this, we will be focusing on a special case of gradient boosting model, which is the Gradient Boosting Decision Tree (GBDT). In this case, each of the models we built like each of these *H*(*X*, −*dL*/*dF*_*n*_(*X*)) would be a tree. There is an interesting part about GBDT; the gamma value, in this case, is calculated at every leaf level. It would be something like that shown in Figure 7. In the figure, each leaf of the tree would have a gamma value.

The article "Detecting Cognitive Impairment Status Using Keystroke Patterns and Physical Activity Data among the Older Adults: A Machine Learning Approach" was published in 2021. Journal: J Healthc Eng.

#### 3.6.2. Support Vector Machine (SVM)

The Support Vector Machine (SVM) [56] is a very popular and widely used algorithm in machine learning for classification and regression [57]. It builds an intricate model as basically as conceivable, so it very well may be effectively investigated numerically. SVM sets aside a less figuring effort to recognize a hyperplane in an *n*-dimensional space (*n* being the number of features) that exclusively groups the information. The current research utilized a Sequential Minimal Optimization (SMO) algorithm with the polynomial piece to upgrade the SVM classifier model. SVM was considered for dealing with the issue of overfitting of high-dimensional information.

### 3.7. Tuning The Model

Our model has been tuned with some hyperparameters to set some customized values to improve our model performance. In this case, we have selected “alpha” to 1.0, “criterion” to friedman_mse. The “n_estimators” is set to 32, which will create 32 DTs within GBM. The “learning rate” is set to 0.1, which determines each tree's impact on the outcome. The “random state” is set to 96; it is a random number seed so that the same random numbers are generated every time. The “colsapmle_bytree” is set to 0.7, which works for random feature selection at the tree. The “max_depth” is to 6; it is a stopping criterion (i.e., a maximum depth to which a tree can grow).

### 3.8. The Model Evaluation and Validation

We have used conventional machine learning algorithms to analyze our participants' neurophysical conditions in this study. We have given accuracy, precision, recall, *F*1-score, and ROC curve; those are employed as evaluation metrics in our experiments to represent our work contribution. We divided our dataset into two parts: two-thirds of the datasets for the training process, and another one-third was for the testing process. To validate the model, we applied 10-fold cross-validation with a 5∗2 approach on the dataset. First, the dataset was divided into two halves randomly. Second, one part was employed in training and another in testing, and we repeated the same procedure as vice versa. This procedure was applied five times repeatedly. Finally, we averaged the results and generated a projected score and compared it with the actual score. This cross-validation procedure has the advantage that all data are used for both validation and training. We have presented a graph comparing the generated score with the actual score in the Results section. The root mean square deviations (RMSDs) have been used to calculate the error between the estimated score (*Ē*_esc_) and the actual score (*Ē*_iesmmse_). The RMSD value defined the model performance and has been calculated as follows:

(16) $$\begin{array}{c} \text{RMSD}=\sqrt{\frac{1}{N}\sum_{i=1}^{N}{\left({\bar{E}}_{\text{iesmmse}}-{\bar{E}}_{\text{esc}}\right)}^{2}.} \end{array}$$

The article "Detecting Cognitive Impairment Status Using Keystroke Patterns and Physical Activity Data among the Older Adults: A Machine Learning Approach" was published in 2021. Journal: J Healthc Eng.

## 4. Results

### 4.1. SMMSE Score Prediction

From participants' neurophysical behavior and physical activities pattern, 11 features have been extracted and divided into three subgroups. The linear regression model has been used to estimate each feature's corresponding cognitive impairment score. According to the cognitive impairment levels' score, four groups have been categorized (normal (SMMSE score ≥ 25), mild (21 ≤ SMMSE score ≥ 24), moderate (10 ≤ SMMSE score ≥ 21), and severe (SMMSE score ≤ 9)). Each subgroup's feature data distribution has a relationship with cognitive impairment symptoms. It has also been found that seven features have a high correlation with cognitive impairment symptoms as their “*p*” values are less than 0.05 to close to 0, as discussed in Section 3.5. These seven features are total time (TT), error number of words (ENW), average time (AVG), absolute energy (AE), quality sleeping time (QST), walking step (WS), and heart pulse data (HPD).

Table 4 represents the relationship between the regression model estimated SMMSE score and the actual score, evaluated using RMSD. The error has been minimized using the lasso regularization method, as discussed in section 3.2.1. Each of the features' results shown in Table 4 is calculated by using leave-one-out cross-validation. A subset has been selected using the wrapper feature selection method among 33 features from three subgroups (base, weekday, and weekend), and this technique shows the lowest RMSD of 3.125. This value demonstrates that the predicted SMMSE score has stronger correlations with the actual SMMSE score.

### 4.2. Cognitive Impairment Level Detection

As shown in Figure 8, data distribution analysis demonstrates that the features are highly distributed, with high standard deviation and too many outliers in features. A rule-based algorithm like “decision trees” or “ensemble learning” should work efficiently for these kinds of feature datasets. In this regard, we have the Gradient Boosting Machine (GBM), an ensemble learning algorithm. For evaluating and proving our selection, we have experimented with a distance-based algorithm, the “support vector machine (SVM)” also.  Table 5 represents the overall accuracy of our used models. We can see that the “gradient boosting machine (GBM)” has the highest accuracy of 94.8%.

The article "Detecting Cognitive Impairment Status Using Keystroke Patterns and Physical Activity Data among the Older Adults: A Machine Learning Approach" was published in 2021. Journal: J Healthc Eng.

In terms of the four cognitive levels—(i) normal, (ii) mild, (iii) moderate, and (iv) severe—the classification algorithm results are shown in Table 6, where classification performance has been demonstrated by showing the results of accuracy of the individual classifier as well as individual classes. We can easily decide on an excellent algorithm to analyze Table 6 as the particular classifier precision, recall, *F*1-score, and accuracy have been given. The accuracy result has shown that GBM generally has done an excellent performance compared with other classification algorithms. In the “normal” class, the SVM accuracy level looks slightly good, but GBM performed well on all four cognitive impairment levels.

The GBM classifier's performance using the receiver operating characteristic (ROC) curve has been shown in Figure 9. As shown in Figure 9, by considering the “normal” cognitive impairment as a negative test sample, the ROC curve in terms of cognitive impairment reached a maximum true positive rate of approximately: (i) 99% for mild cognitive impairment, (ii) 96% for severe cognitive impairment, and (iii) 94% for moderate cognitive impairment. In Figure 10, we have shown the random 15-day data of our participants for every cognitive impairment class. This figure demonstrates and validates the accuracy of the model. The mild (21 ≤ SMMSE score ≥ 24), moderate (10 ≤ SMMSE score ≥ 21), and severe ( SMMSE score ≤ 9) levels have a range, and if the value is within range, we have counted as an actual prediction, otherwise false prediction.

## 5. Discussion

This study used keystroke pattern data and smart wearable device data to extract information about our participants' neurophysical behavior and physical behavior patterns. We have used the “10-fold-cross-validation” with a 5∗2 approach to validate our model. The model can detect four different cognitive impairment levels (i.e., normal, mild, moderate, and severe) with 94.8% accuracy. This accuracy is higher than that in a previous study, which recorded an accuracy rate of 86% [58]; however, this study focused on predicting dementia and mild cognitive impairment. Our extracted features from our developed application and wearable devices data have shown a strong correlation with the SMMSE score and are found in the regression model.

The article "Detecting Cognitive Impairment Status Using Keystroke Patterns and Physical Activity Data among the Older Adults: A Machine Learning Approach" was published in 2021. Journal: J Healthc Eng.

The study by Vizer and Sears [28] was based on typed text's keystroke and linguistic features to detect cognitive impairment. Some researchers like Sofi et al. [59] did a meta-analysis on physical activity. In the present study, we have combined keystroke pattern behavior with our participants' physical activity to detect cognitive impairment.

In our study, using the “Pearson” correlation for feature analysis and wrapper method to select the features has done a great job to achieve higher accuracy classification performance for each cognitive impairment level (normal, mild, moderate, and severe). To evaluate the classification performance, we have used two popular classification algorithms: GBM, SVM, and the GBM have shown better performance and higher accuracy in every cognitive level.

*Limitations*. Although the model used in this research predicted cognitive impairment level with high accuracy, there are some limitations when interpreting the results. This research did not assess a clinically cognitive impaired population because the sample only comprised older adults. The assessment used to evaluate cognitive impairment was a self-report scale called the SMMSE rather than a clinical evaluation. Typing errors, taking a long time to complete sentences, or being unable to remember words might be critical factors for cognitive impairment. Some physical issues can be related to what this research tried to find out. But noncognitive impaired people might have those same problems for several reasons. Besides, some participants may not have followed our instructions carefully, which would make some data errors. Like answering misconceptions, participants may not always wear smartwatches, etc.

## 6. Conclusions

Machine Learning (ML) innovation holds noteworthy guarantees for changing how we determine and treat patients with neurocognitive disorders. There exists an enormous assortment of potential highlights that in a mix can exhaustively describe the biopsychosocial determinants of an exceptional individual and consequently empower a more customized comprehension of intellectual decay. ML calculation presentation and potential clinical utility for distinguishing, diagnosing, and predicting psychological decline utilizing these highlights will keep on improving as we influence multifeature datasets on massive datasets. Setting up rules for research, including AI applications in medical services, will be essential to guarantee the nature of results and clinicians' commitment, besides allowing patients and their caregivers to contribute their ability to refine AI calculations. This study demonstrated the capability to passively detect cognitive impairment symptoms by monitoring daily physical activities and keystroke patterns. Given that the detection of cognitive impairment level is not dependent on traditional self-report psychometric instruments, such a method may improve the identification of cognitive impairment. Early detection of these progressions can allow for interventions that can lessen, delay, or thwart related functional impairments. Therefore, more effective techniques that support the early detection of cognitive changes, mostly solutions that continuously leverage normal daily activities, could significantly impact older adults' health and independence. Given the connection between cognitive processes expected to utilize innovation and those affected by cognitive impairment and stress, this examination will investigate keystroke and physical attributes of unexpectedly composed content as a potential methodology for checking cognitive changes. This methodology has a few points of interest over conventional techniques for observing cognitive function. Therefore, the proposed model in this study can examine the totality of the data not just at specific stages. It is subtle and assembles standard information for examination and finding just as constant information for everyday monitoring.

The article "Detecting Cognitive Impairment Status Using Keystroke Patterns and Physical Activity Data among the Older Adults: A Machine Learning Approach" was published in 2021. Journal: J Healthc Eng.

## Figures and Tables

**Figure 1:** The graphical abstract of research planning. (a) Data acquisition. (b) Data preprocessing and analyzing features. (c) Machine learning approach. (d) Result analysis.

**Figure 2:** The distribution of datasets between original data and augmented data.

**Figure 3:** Correlation matrix heatmap with “*r*” values of features.

**Figure 4:** Correlation matrix heatmap with “*p*” values of features.

**Figure 5:** The “GBM” model working procedure steps.

**Figure 6:** The “GBM” mathematical modeling block.

**Figure 7:** The “GBDT” block with gamma value in the leaf.

**Figure 8:** The distribution of values of the dataset. Features values have been normalized between 0 and 1 and the interquartile range (IQR) in the box between 25% and 75%. The median line 50% of the values of the features falls between 25% and upper 75%, and the “+” sign represents outliers of features.

**Figure 9:** The ROC curve demonstrates the performance of the classification of each cognitive impairment level. The yellow curve (mild cognitive impairment) shows higher performance, while the red curve (severe cognitive impairment) has a little bit lower result, and the blue (moderate cognitive impairment) shows lower performance.

The article "Detecting Cognitive Impairment Status Using Keystroke Patterns and Physical Activity Data among the Older Adults: A Machine Learning Approach" was published in 2021. Journal: J Healthc Eng.

**Figure 10:** Comparison between the actual score and the projected score of model. (a) Mild. (b) Moderate. (c) Severe.

**Table 1:** SMMSE scores of the participants.

	SMMSE score ≤ 9	10 ≤ SMMSE score ≥ 21	21 ≤ SMMSE score ≥ 24	SMMSE score ≥ 25
Participants	2	3	6	22
Cognitive impairment	Severe	Moderate	Mild	Normal
Gender	One male; one female	Two males; one female	Four males; two females	19 males; three females
Age ± SD	64 ± 1	60 ± 2	56 ± 1	52 ± 2
No. of months activity recorded	6	6	6	6

**Table 2:** Dataset sample.

Application data				Wearable device data							Group
TNW	TT (sec)	ENW	AVG (sec)	AE (kcal)	QST (hour)	WS	St (hour)	HPD	DC (metre)	CT (hour)	Class
10	8	1	1.33	305.5	7	650	10	84	1400	1.5	0 (N)
12	10	2	1.66	240.67	8	755	12	78	1800	2.5	1 (MCI)
8	7	1	1	332.5	6	750	9	65	1200	2	3 (S)
15	12	2	2	357.5	5	595	10	73	1500	1.25	2 (M)
13	10	3	1.67	190.87	7	580	11	79	1300	3	3 (S)

**Table 3:** Participants' neurophysical and physical activity features.

Feature	Abbr.	Extraction process
Total number of words	TNW	Ēt*nw* represents t0068e total number of words in a complete sentence. In the formula, the user-given sentence's total number of words is represented by *Wn*. The total number of word parameters is acquired using our application, developed for this study. Ēt*nw* = *W*1 + *W*2+...+*Wn*
Total time	TT	Ēte represents total time. In the formula, user taken time is represented by *Tt*. The total time parameters are acquired using our application, developed for this study. Ēte = *Tt*
Error number count of word	ENW	Ē represents the calculated error number count of words parameter. In the formula, *E*_*nw*_ indicates an error count of the current iteration. *Ē*_*ec*_ is the current calculated value of error count, and *Ē*_*ec*_− 1 is the previously calculated value of the error count. The error number count of word parameters is acquired using our application, developed for this study. *Ē*_*ec*_ = $\left({\bar{E}}_{ec}-\;1+E_{nw}\right)/2$
Average time	AVG	*S*_*l*_ represents sentence length. *Ē*_*te*_ represents total time. AVG = ${\bar{E}}_{te}/S_{l}$
Absolute energy	AE	Energy is assessed in two main parts: active energy (eae) and rest (ere) energy. Ēem is a representation of absolute energy in the given formula. The energy parameter is acquired using a smartwatch daily basis. Ēem = eae + ere
Quality sleeping time	QST	Based on the National Sleep Foundation's professional's research, an age-specific sleep duration recommendation is called Sleep Health Index (SHI) [52]. Ēqst identifies the quality sleeping timing parameter. It is a consistent incentive for every day, relying upon sleep time. The quality sleeping time parameter is acquired using a smartwatch daily basis. Ēqst = Qst
Walking steps	WS	Walking steps (ews) value was taken for a period of time. Ēws stands for walking steps parameter, which is the sum of the incremental steps over the day. The walking steps quantity parameter is acquired using a smartwatch daily basis. Ēws = ews
Sitting time	ST	The sitting time (est) value was taken while the participant was in an idle mood and not sleeping. Ēst stands for sitting time parameter, which is the sum of the different idle periods over the day. The sitting time parameter is acquired using a smartwatch daily basis. Ēst = est
Heart Pulse data	HPD	The average heartbeat value is denoted as the base heartbeat value (*H*_*b*_). All base and abnormal heartbeats (*H*) are calculated, and the average value of heartbeats is calculated for each hour. The daily value is calculated as the average value of hourly values. This heart pulse parameter is acquired using a smartwatch hourly. Ēhb = (*H*_*b*_+∑_*k*=0_^*n*^*H* )/(*n*+1)
Distance Covered	DC	Distance covered (edc) value was taken while the participant was running. Ēdc stands for distance covered parameter, representing how long the participant was running over the day in the hour's scale. The distance covered parameter is acquired using a smartwatch daily basis. Ēdc = edc
Cycling time	CT	Cycling time (ect) value was taken while the participant was cycling. Ēct stands for cycling time parameter, representing how long the participant was cycling over the day in the hour's scale. The cycling time parameter is acquired using a smartwatch daily basis. Ēct = ect

The article "Detecting Cognitive Impairment Status Using Keystroke Patterns and Physical Activity Data among the Older Adults: A Machine Learning Approach" was published in 2021. Journal: J Healthc Eng.

**Table 4:** The error rate between the actual score and the estimated score.

Feature	Base subgroup	Weekday subgroup	Weekend subgroup	Wrapper selected features
TNW	5.102	4.795	4.988	3.125
TT	4.112	4.256	4.394	
ENW	4.226	4.129	4.186	
AVG	4.274	4.202	4.195	
AE	4.245	4.195	4.113	
QST	4.114	4.052	4.123	
WS	4.218	4.253	4.209	
ST	5.044	4.725	4.826	
HPD	4.032	4.107	3.975	
DC	5.096	4.923	4.753	
CT	5.077	4.889	4.662	

**Table 5:** Summary of overall classification accuracy.

Classifier name	Accuracy (%)
Gradient boosting machine (GBM)	94.8
Support vector machine (SVM)	61.5

**Table 6:** Summary of classification results.

Cognitive level	Classifier	Precision (%)	Recall (%)	*F*1-score (%)	Accuracy (%)
Normal	GBM	92.2	99.2	95.5	96.6

	SVM	80.1	94.4	87.7	87.8

Mild	GBM	93.3	99.2	96.5	97.7
	SVM	49.9	40.1	44.4	45.5

Moderate	GBM	89.1	90.2	87.8	91.1
	SVM	64.5	48.5	54.5	56.6

Severe	GBM	91.1	92.2	88.2	94.4
	SVM	64.5	49.9	55.5	58.7

## Data Availability

The datasets in this study are collected from users as a part of this study. Thus, these can be shared upon request.
